# Significance of the Asymmetry of the Haltere: A Microscale Vibratory Gyroscope

**DOI:** 10.1155/2020/8647137

**Published:** 2020-11-17

**Authors:** Rizuwana Parween

**Affiliations:** Mechanical Engineering Department, Indian Institute of Science, Bangalore, India

## Abstract

Nature has evolved a beautiful design for small-scale vibratory gyroscopes in the form of halteres located in the metathorax region of the dipteran flies that detect body rotations based on the Coriolis principle. The specific design of the haltere is in contrast to the existing MEMS vibratory gyroscope, where the elastic beams supporting the proof mass are typically designed with symmetric cross-sections so that there is a mode matching between the actuation and sensing vibrations. The mode matching provides high sensitivity and low bandwidth. Hence, the objective of the manuscript is to understand the mechanical significance of the haltere's asymmetry. In this study, the distributed Coriolis force and the corresponding bending stress by incorporating the actual mass variations along the haltere length are estimated. In addition, it is hypothesied that sensilla sense the rate of rotation based on the differential strain (difference between the final strain (strain due to the inertial and Coriolis forces) and the reference strain (strain due to inertial force)). This differential strain always occurs either on the dorsal or ventral surface of the haltere and at a distance away from the base, where the campaniform sensilla are located. This study brings out one specific feature—the asymmetric geometry of the haltere structure—that is not found in current vibratory gyroscope designs. This finding will inspire new designs of MEMS gyroscopes that have elegance and simplicity of the haltere along with the desired performance.

## 1. Introduction

Angular rate sensors (gyroscopes) are one of the primary components in inertial navigation systems (INS), virtual reality products, and some consumer electronic devices for measuring the rate of rotation. Based on the operating principle, there are four basic types of gyroscopes: classical (spinning mass or rotary), optical, solid-state ring lasers, and vibratory mass gyroscopes [1]. Over the last two decades, MEMS (microelectromechanical system) vibratory gyroscopes have been developed and made commercially available due to the evolution of the microsystem technology. They exploit Coriolis acceleration for sensing rates of rotation.  Figure 1(a) shows the 3D view of a simple MEMS vibratory gyroscope that consists of a large proof mass structure suspended with four flexural beams. The suspension system consists of long prismatic beams of rectangular cross-section that help in oscillation of the proof mass. The flexible suspension system is actuated by an electrostatic force of frequency equal to the natural frequency along the drive direction (*x*-axis) to facilitate resonance-driven large-amplitude motion. In response to an angular rotation in the *xy* plane (i.e., about the *z*-axis), applied to the gyroscope, Coriolis force gets induced which makes the proof mass oscillate at the actuation mode frequency in the sense direction (*y*-axis). The induced Coriolis force deflects the proof mass along the sensing direction, and this deflection is sensed by the sense electrodes.

In 1993, Greiff et al. from Draper Lab of MIT developed the first MEMS vibratory gyroscope [2] as shown in Figure 1(b). This gyroscope had a double-gimbal silicon structure connected by torsional flexural beams, which employed electrostatic actuation and capacitive sensing. As the vibratory gyroscopes must have an oscillating or vibrating structure for sensing the rate of rotations, the research community looked at various other designs such as beams [3], rings [4], tuning forks [5], and spinning disks [6] as vibrating structures. The main issues associated with these MEMS gyroscopes are complexity in the design, system level integration, and packaging techniques. They are packaged under vacuum condition. If there is any leakage or faulty packaging, the pressure and temperature levels fluctuate, affecting the operation of the gyroscope severely. The fabrication of MEMS gyroscopes also involves complicated techniques that significantly affect the final released structure and material properties by inducing residual stresses, which degrade the performance of the device. Therefore, the dynamical system characteristics of this device are very susceptible to the fabrication process and packaging conditions. Therefore, there is a need to look for alternative designs and fabrication techniques for gyroscopes which can be produced in high volume. The research community is trying to get inspirations from nature's design in order to overcome the above constraints.

Nature has developed an elegant design of microscale vibratory gyroscope operating based on Coriolis principle called halteres, used by dipteran insects [7]. They provide the feedback about the rates of rotation to the wing during aerial maneuver.  Figure 2(a) shows the haltere of a soldier fly, *Hermetia illucens* (dipteran fly). Each haltere consists of a long stalk with a massive end knob and distinct fields of mechanosensory organs called campaniform sensilla at the base as shown in Figures 2(b) and 2(c). During maneuver, any rotation of their body (pitch, yaw, or roll) results in a microscale out-of-plane motion of the halteres due to the induced Coriolis force. The resulting deflection at the haltere base is very small, and the halteres use specialized mechanosensory organs (sensilla at the base) to sense this tiny deflection. These sensilla convert the mechanical deflection of the haltere to a neuronal signal, and the fly's nervous system decodes the neural signal to figure out the rate of rotation.

In contrast to the MEMS gyroscopes, the halteres follow a completely different design principle. Firstly, the MEMS gyroscope has a single sensing element to sense the Coriolis force-induced out-of-plane deflection. However, it has been studied by a few groups of researchers that the fields of campaniform sensilla act as strain sensors [8], and haltere-inspired gyroscopes were developed. Droogendijk et al. developed a gimbal-suspended gyroscope inspired by the fly's haltere using microelectromechanical system (MEMS) technology which showed a large measurement bandwidth and a fast response [9, 10]. Smith et al. designed and fabricated a novel IMU based on the biological haltere system in a microelectromechanical system with a developed efficient control scheme that efficiently and accurately decouples the three component parts from the haltere sensors [11]. Kilic et al. developed an optoelectromechanical vibratory gyroscope inspired by halteres of dipteran flies. The gyroscope utilizes optical displacement sensing to achieve Brownian motion-limited displacement sensitivity without mechanical resonant amplification in the sense mode [12]. Chen et al. presented and discussed the preliminary design of a new bioinspired surface micromachined MEMS vibratory gyroscope [13].

Figure 3 shows the scanning electron microscopy (SEM) images of the dorsal and ventral surfaces of the soldier fly's haltere base with a few distinct fields of sensilla. Pringle classified these mechanosensory sensilla into two groups: the campaniform sensilla and chordotonal organs [7]. There are three distinct fields of sensilla (basal plate, scapal plate, and Hick's papillae) on each dorsal and ventral surface, and a large chordotonal organ at the base, shown in Figure 4. Pringle laid a theoretical basis for the function of each sensillum field and mentioned that the basal plate and the large chordotonal organs are responsible for sensing the Coriolis force [7]. Till today, there is no experimental evidence of the distinct functions of each sensillum field. Therefore, the distribution and arrangement of these sensilla at the haltere base are important aspects of the fly's sensing mechanism. Secondly, in the case of MEMS gyroscopes, due to the same natural frequency in both directions, there is a maximum energy transfer between the actuation and sensing modes and the deflection along the sensing direction is maximum. This behavior is called frequency or mode matching. The frequency matching between the actuation and sensing modes increases the sensitivity of the gyroscopic system. The haltere has a larger amplitude of motion as compared to the MEMS vibratory gyroscopes. In our previous work, Parween and Pratap presented the stiffness of the haltere along both the actuation and sensing directions [14]. The natural frequency along the sensing direction was found to be higher than the natural frequency along the actuation direction.

The fly relies on the halteres for quicker flight stability as they provide faster feedback signal during maneuvers [15–17]. The halteres enhance the stability of the body during any undesirable self-perturbation or any environmental disturbances such as airflow. Even though both halteres are coupled and controlled by the fly's nervous system, they can decouple the complex rotations very efficiently [18]. They are exposed to air and operate in the normal atmospheric conditions without any special packaging system.

The haltere represents a cantilevered structure which is simple in design as compared to the existing classical and MEMS vibratory gyroscopes [7]. Each haltere consists of a long-tapered stalk of elliptical cross-section. This implies that the haltere has asymmetry along the length and the cross-section as well (MEMS Gyro have symmetric design). As compared to the MEMS vibratory gyroscopes, it has not yet been established if the haltere's asymmetry induces any valuable effect on any of its gyroscopic performances (sensitivity, bandwidth, or sensillum location). In the previous work, a model of the haltere's actuation and sensing mechanisms was considered and the effect of the gyroscopic force during three orthogonal rotations (pitch, yaw, and roll) on the stress pattern at the haltere base was presented. The stress pattern did not include any effect of inertial force. The finite element analysis was carried out on the simplified haltere model (a cylindrical stalk with a spherical knob). The variation of the haltere's cross-section was not considered. However, in this paper, an attempt was made to uncover the underlying mechanics rationale behind the distribution of the sensilla at the haltere base considering the inertial force and haltere's asymmetry.

From mechanics, it is known that any cantilever beam undergoes the maximum bending stress at the base. If at all the campaniform sensilla sense the maximum stress caused due to the out-of-plane bending deformation of the haltere, then they have to be located at the base. However, the campaniform sensilla on both the dorsal and ventral surfaces are located somewhat away from the base. It is suspected that the haltere's asymmetry is correlated with the sensillum location on the dorsal and ventral surfaces. These facts about the haltere's design motivate me to study the following aspects about the asymmetry of the haltere: (1) Why do halteres have asymmetry along both the length and the cross-section? (2) Why are the sensilla located away from the base?

## 2. Material

Two-day-old, laboratory-reared soldier flies (*Hermetia illucens*) were collected and anesthetized by cooling in the refrigerator at 4°C for 10 minutes, and then the samples were prepared as per the requisites of the imaging techniques. In order to know the haltere's geometry, the haltere specimen was dissected from the anesthetized soldier fly and kept on a thin sheet ruled with grids, with grid spacing of 0.25 mm, and the images of the haltere were taken by keeping them along the dorsal side.

## 3. Haltere Mechanics

The fly flaps its halteres in the flapping plane, inclined at an angle 30° with its transverse axis (*T*), shown in Figure 5(a). Each haltere oscillates at a particular frequency with a large amplitude (170°) in the flapping plane as shown in Figure 5(b). The large amplitude of the haltere helps in amplifying the Coriolis force. Due to the nonorthogonality of the haltere's flapping planes, dipteran flies can measure the body rotations during hovering, roll, pitch, and yaw movements [19, 20].  Figure 6 shows the cross-section of the thorax along the haltere's flapping plane. *m* is the mass of the haltere acting at its center of mass “*C*”. The flapping plane along with the connecting joint at “*o*” (where the haltere is attached to the fly's body) represents the body frame. $\vec{r}$, $\vec{v}$, and $\vec{a}$ are the position, velocity, and acceleration, respectively, of the center of mass relative to “*o*”. When the insect does not undergo any translational or rotational motion, due to the haltere's flapping, the inertial force ($m\vec{a}$) and gravitational force (*mg*) act on it. However, when the fly's body rotates about different axes (pitch, yaw, and roll), apart from these gravitational and inertial forces, a few additional forces act on the haltere. Let $\vec{\Omega }$ and $\vec{\dot{\Omega }}$ be the angular velocity and angular acceleration of the insect's body with respect to the inertial frame, respectively. As a result of the insect body rotation and haltere's flapping, the net force ($\vec{F}$) acting on the haltere is $\vec{F}=m\vec{a}+mg+m\vec{\Omega }\times \left(\vec{\Omega }\times \vec{r}\right)+2m\left(\vec{\Omega }\times \vec{v}\right)+m\left(\vec{\dot{\Omega }}\times \vec{r}\right)$, where $m\vec{\Omega }\times \left(\vec{\Omega }\times \vec{r}\right)$, $2m\left(\vec{\Omega }\times \vec{v}\right)$, and $m\left(\vec{\dot{\Omega }}\times \vec{r}\right)$are the centrifugal force, Coriolis force, and tangential acceleration force, respectively.

In 1993, Nalbach estimated the magnitude of each force based on the haltere's experimentally observed velocity and acceleration along the trajectory and estimated the relative magnitudes of the forces acting on the haltere analytically. Based on his estimates, he reported that the Coriolis forces were the predominant force among other components of force that contains information on the axis, sign, and velocity of the insect's body rotation. He showed that primary inertial force provided the biggest contribution to the total force. Sandeman claimed that it is possible for the halteres to detect the insect's acceleration from the angular acceleration force. However, the angular acceleration-dependent force is much smaller than the Coriolis force, and it is observed that in flapping frequency up to 50 Hz, the acceleration term is less than one-fifth of the Coriolis force [21]. Thus, the halteres were established as vibratory rate gyros that detect the rate of rotation of the fly's body during aerial rotations (pitch, yaw, and roll).

## 4. Significance of Sensillum Location

The presence of the sensilla at the haltere base implies that the strain at any point on the haltere base is a primary sensing signal. These sensilla act as strain gauges that decode the primary strain signal into the rates of rotation. In this section, the haltere model was considered a cylindrical stalk with a spherical end mass, with fixed boundary conditions at the base. The inertial force and Coriolis force due to the pitch, yaw, and roll rotations of the fly and the corresponding elastic strain (strain due to the Coriolis force and inertial force) variation along the periphery of the cross-section were estimated. Based on the dimensions, the mass of the haltere stalk was obtained which is as an order of magnitude smaller than the end mass. Thus, for strain estimates, the Coriolis force on the haltere stalk was ignored and the Coriolis force acting on the end mass alone was considered at any generic position during the upstroke and downstroke directions. Next, the analytical strain by carrying out finite element analysis (ANSYS) with the analytically obtained Coriolis force was verified.

Figure 7(a) shows the dorsal view of the fly in the *XZ* (midsagittal) plane with the abdomen pointing along the *Z*-axis. The *X*- and *Z*-axes represent the transverse and longitudinal axes of the fly, respectively. The rotations about the *X*-, *Y*-, and *Z*-axes indicate the pitch, yaw, and roll rotations, respectively. The right haltere at an angle *β* (30°) with respect to the *X*-axis such that the longitudinal axis of the haltere passes through the point *O* was considered. Another *xyz* coordinate system at point *O*, with the *x*-axis along the longitudinal axis of the haltere stalk, was included.  Figure 7(b) shows the haltere stalk of length *L* with a knob of radius *d* and mass *m* oscillating at its natural frequency *f*_*d*_ in the actuation plane (*xy* plane). A polar coordinate system (*e*_*r*_, *e*_*θ*_, and *e*_*z*_) at the mass center of the knob that oscillates with the haltere was added. The haltere is approximated as a cylindrical stalk with a spherical end knob shown in Figure 7(c).

A generic position *P* of the end knob, at an angle *θ* with the *x*-axis in the actuation plane (both the upward and downward strokes), is considered as shown in Figure 8. The position vector of the center of mass of the right haltere is (*L* + *r*)*e*_*r*_. The angular position of the right haltere in the actuation plane follows *θ* = *θ*_*m*_sin(*ω*_*d*_*t*), where *ω*_*d*_(2*πf*_*d*_) is the angular frequency along the actuation direction. The angular velocity of the right haltere is *θ* = *θ*_*m*_*ω*_*d*_cos(*ω*_*d*_*t*)*k*. The tangential velocity of the right haltere is *v* = *θ* × *r* = *θ*_*m*_(*L* + *d*)*ω*_*d*_cos(*ω*_*d*_*t*)*e*_*θ*_. For an angular rotation *Ω* about the *X*-axis (pitch rotation), the Coriolis force acting on the right haltere is

(1) $$\begin{array}{c} F_{\text{CP}}=2m\Omega I\times v=A\left(\cos\beta \cos\theta e_{z}+\sin\beta e_{r}\right), \end{array}$$

where *A* = 2*mΩθ*_*m*_(*L* + *d*)*ω*_*d*_cos(*ω*_*d*_*t*). Similarly, the Coriolis force on the right haltere when the fly rotates about the *Y* (yaw) or *Z* (roll) axis is estimated, as given in Table 1. The strain at the *Q* point due to the pitch rotation is given by

(2) $$\begin{array}{c} \epsilon_{rr}=\frac{A\sin\beta }{E\pi r^{2}}+\frac{A\cos\beta \cos\theta \left(L+d\right)a\cos\eta }{EI}. \end{array}$$

The angular speed as 10 rad/sec during the pitch rotation and the amplitude of oscillation as 85° along the actuation direction were considered. Let the length (*L*) of the stalk, radius (*a*) of the stalk, and radius (*d*) of the end knob be 1000 *μ*m, 11 *μ*m, and 220 *μ*m, respectively. From the literature, the density of the haltere material is taken as 1200 kg/m^3^ [22] and Young's modulus of the haltere as 625 MPa [14, 23]. By using these data, the elastic strain at four points A, C, B, and D on cross-section during the upstroke and downstroke was estimated.  Figure 9(a) shows the strain variation across the cross-section during the upstroke motion of the haltere for the pitch, yaw, and roll rotations. We observe that the maximum strain occurs at C for any rotation.  Figure 9(b) shows the strain variation across the cross-section during the downstroke motion of the haltere. During the downstroke motion of the haltere, the maximum strain occurs at A, due to any rotation.  Figure 10 shows the strain variation across the cross-section during upstroke due to different rotations obtained from the FE simulations. It also shows that the maximum strain due to Coriolis force always occurs irrespective of the rotation, which is in agreement with the analytical result.

When the haltere flaps in the actuation plane, the haltere experiences inertial force. As the inertial force is independent of the fly's body rotation, the halteres are always subjected to this force even if the fly does not rotate. Therefore, the inertial force and the corresponding strain generated at the haltere base were estimated by using finite element simulation. The inertial force has two components, i.e., radial and tangential. The radial component of the inertial force is given by

(3) $$\begin{array}{c} \vec{F_{r}}=m\vec{\dot{\theta }}\times \left(\vec{\dot{\theta }}\times \vec{r}\right)=-m\left(L+d\right){\left(\theta_{m}\omega_{d}\cos\omega_{d}t\right)}^{2}e_{r}, \end{array}$$

The tangential component of the inertial force is given by

(4) $$\begin{array}{c} \vec{F_{t}}=m\vec{\ddot{\theta }}\times \vec{r}=-m\left(L+d\right)\theta_{m}{\left(\omega_{d}\right)}^{2}\sin\omega_{d}te_{\theta }. \end{array}$$

Equations (3) and (4) show that the radial and tangential components of the inertial force always act along the *e*_*r*_ and *e*_*θ*_ directions, respectively. At position *P* (during upstroke), by estimating the radial component and tangential component of the inertial force and by applying these forces to the model, a finite element analysis was carried out to obtain the combined strain generated at the haltere base due to pitch rotation.  Figure 8(a) shows the strain pattern across the cross-section of the haltere base due to the inertial force.  Figure 8(b) shows the combined strain pattern due to 10 rad/sec.

## 5. Significance of the Haltere's Asymmetry

In order to understand the significance of the haltere's asymmetry, two different models of the haltere are created using (1) accurate external features and (2) both external and internal features. In the first case, the mass variations along the haltere length by using external geometrical features (solid cross-section) were considered and the distributed Coriolis force and the corresponding stress were estimated analytically. Then, the variation of the stress along the length due to the Coriolis and inertial forces was figured out. In order to verify the analytical result, a three-dimensional structural haltere model with a solid cross-section throughout the length was considered. By applying the inertial and Coriolis forces, FE analysis was carried out in ANSYS. In the second case, a three-dimensional detailed haltere model by incorporating all the external and internal geometrical features (hollow cross-section) was carried out and a finite element simulation was performed to estimate the stress variation across the length.

### 5.1. Haltere Model with Accurate External Features

Figure 11 shows the image of the haltere along the dorsal and lateral sides. In the lateral side image, there is not much variation in the depth *h* along the *y*-axis; the variation in width along the length was considered. In the dorsal image, a reference line *L*_1_ was drawn which is horizontal to the upper bounding line. In order to get the width variation *b*(*r*) along the *z*-direction, several points on the *L*_2_ line was considered; their coordinates were extracted by using ImageJ software. By fitting a polynomial curve along those points, the width variation along the haltere's length was obtained.

In the curve fitting as shown in Figure 12, the variation in width was obtained as follows: the relation *b*(*r*) = 16.35*r*^6^ − 54.8*r*^5^ + 70.8*r*^4^ − 45*r*^3^ + 13.5*r*^2^ − 1.17*r* − 0.267.

Next, the differential element at a distance *r* was considered assuming the density *ρ* to be constant throughout the haltere length, and the Coriolis and inertial forces on the differential element were estimated.-. The area (*dA*), volume (*dV*), and mass (*dM*) of the differential element are given by *πb*(*r*)*h*, *πb*(*r*)*hdr*, and *πρb*(*r*)*hdr*, respectively. The Coriolis acceleration acting on the differential element due to the pitch rotation is given by

(5) $$\begin{array}{c} a_{\text{Pitch}}=2\Omega r\theta_{m}\omega_{d}\cos\omega_{d}t\left(\cos\beta \cos\theta e_{z}+\sin\beta e_{r}\right). \end{array}$$

The Coriolis force on the differential element *dr* is given by

(6) $$\begin{array}{c} dF=dma_{\text{Pitch}}=\pi \rho b\left(r\right)hdr2\Omega r\theta_{m}\omega_{d}\cos\omega_{d}t\left(\cos\beta \cos\theta e_{z}+\sin\beta e_{r}\right)=Arb\left(r\right)dre_{z}+Brb\left(r\right)dre_{r}, \end{array}$$

where *A* = 2*πρhΩθ*_*m*_*ω*_*d*_cos*ω*_*d*_*t*cos*β*cos*θ* and *B* = 2*πρhΩθ*_*m*_*ω*_*d*_cos*ω*_*d*_*t*sin*β*.

At any particular time instant, *A* and *B* are constants, and therefore, the Coriolis force is a function of *r* only. The Coriolis forces along the *e*_*z*_ and *e*_*r*_ directions produce bending stress and axial stress along the *e*_*r*_ direction. The force per unit length along the *e*_*z*_ direction is given by $\vec{q}=Arb\left(r\right)$. The bending moment ($\vec{M}$) on the differential element can be obtained from $d^{2}\vec{M}/dr^{2}=-\vec{q}$. The section modulus on the differential element of solid cross-section throughout the length is given by *Z*(*r*) = *αb*(*r*)^2^*h*, where *α* is a constant. The longitudinal bending stress and the axial stress components acting on the differential element along the *e*_*r*_ direction are given by *σ*_*b*_ = *M*(*r*)/*Z*(*r*) and *σ*_*a*_ = *Brb*(*r*)*dr*/*πVb*(*r*)*h*, respectively. The total bending stress along the *e*_*r*_ direction is given by *σ*_*rr*_ = *σ*_*b*_ + *σ*_*a*_. The variation of the total bending stress along the length of the haltere is shown in Figure 13(a). The result shows that the maximum bending stress occurs at a distance 0.42 mm from the base.

A three-dimensional structural haltere model was constructed with a solid cross-section throughout the length to verify the analytical result. In the previous section, it was claimed that the differential strain stimulates the sensilla and the significance of the location of the sensilla on the dorsal and ventral surfaces in the context of the gyroscopic strain distribution was discussed.  Figure 13(b) shows the variation of the total bending stress along the haltere length, obtained from the finite element simulations. The stress was found to be maximum at the thinnest section, which is at a distance 0.44 mm from the base. The finite element result is in good agreement with the analytical result. However, the sensilla are not at the thinnest cross-section. They are located in between the base and the thinnest cross-section of the stalk.

### 5.2. Haltere Model with Accurate External and Internal Features

To get the cross-sectional details of the halteres, the haltere was dissected at three critical regions (the base, stalk, and knob), and the respective samples were prepared. The SEM images are shown in Figure 14 [13]. The knob is a massive part with a solid cross-section. The haltere stalk is composed of two different tubular structures attached to each other. The thickness values of the haltere stalk and the intermediate joining wall in the stalk are 15 *μ*m and 20 *μ*m, respectively. For creating the three-dimensional structural model of the haltere, the intermediate wall was not considered. The stalk was considered to be a hollow structure of wall thickness 15 *μ*m. The cross-section at the base of the haltere was found to be a tubular structure of thickness 10 *μ*m. Using the image processing software called ImageJ, the size of each pixel of the scale bar given in the image and the dimensions of the haltere's width and depth at various sections were estimated. In ANSYS Workbench, the cross-sections at various haltere lengths were constructed through “skin command” [13]. The inertial and Coriolis forces were applied, and the bending analysis was carried out in ANSYS. The stress pattern is shown in Figure 15. The figure shows that the maximum stress occurs near the base but neither at the base nor at the thinnest section.

## 6. Discussions

### 6.1. Significance of Sensillum Location on the Periphery

In order to find the significance of sensillum location on the haltere base, we have modeled the haltere as a simple cantilevered structure and determined the nature of the combined strain arising across the cross-section due to the Coriolis and inertial forces during various insect body rotations (pitch, yaw, and roll). The results show the Coriolis force produced due to the rotation about the pitch and roll axes is a combination of axial force (along the *e*_*r*_ direction) and flexural force (along the *e*_*z*_ direction). However, during the yaw rotation, the Coriolis force is only along the *e*_*z*_ direction. Analysis shows that the Coriolis force has components along either *e*_*z*_ or *e*_*r*_ or both directions. Both analytical and simulation results show that the maximum strain due to the Coriolis forces occurs on the side surfaces of the haltere (at C during upstroke motion and at A during downstroke motion of the haltere) for any rotations. Since at any instant during an aerial rotation both the inertial and Coriolis forces act on the haltere, the strain due to inertial force as well needs to be considered. This combined stress due to the effect of the Coriolis and inertial forces causes maximum strain at B, the dorsal surface of the haltere during upstroke motion.

Simulations were carried out for both the slower and faster rotations of the haltere. In both cases, the maximum combined strain occurs at B during upstroke, where the campaniform sensilla are located. The magnitude of the combined strain during slow angular rotation is the same as that of the strain due to the inertial force. It is because, during slow angular speed, the magnitude of the inertial force is higher than the magnitude of the Coriolis force. As a result, the inertial force has a dominant effect on the location and the magnitude of the maximum strain. During fast angular speed, a substantial difference between the magnitude of the combined strain and the inertial strain was found. However, in both cases, during the upstroke motion, the location of the maximum strain due to the combined strain occurs at B (dorsal surface), where the sensilla are located. Similarly, during downstroke, the maximum strain occurs at D (ventral surface).

If at all any field of the campaniform sensilla senses the maximum strain due to the Coriolis force, then the sensilla should be located on the side surfaces. However, the sensilla are located on the dorsal and ventral surfaces, not on the side surfaces. It shows that the sensilla cannot detect the maximum strain due to the Coriolis force. Then, it is wondered how the campaniform sensilla sense the strain due to the Coriolis force-induced bending of the haltere during the aerial rotations. This issue is addressed by incorporating the strain arising due to the inertial force.

It is observed that the location of the maximum combined strain is independent of the angular speed (slow or fast) and it always occurs at either the dorsal or ventral surface. If at all the sensilla senses the combined strain induced due to both the inertial and Coriolis forces, then how they detect the rate of rotation as the inertial force does not contain any information about the rate of body rotation. Based on the above observation, it is proposed a simple strain sensing mechanism. The inertial force produces maximum strain on the dorsal surface, where the campaniform sensilla are located. The inertial strain stimulates these sensilla. The sensilla keep this strain (strain due to inertial force) as the reference strain. When the fly rotates its body, the strain due to Coriolis force gets superimposed on the reference strain and the sensilla measure the differential strain. The differential strain is considered the difference between the final strain (strain due to the inertial and Coriolis forces) and the reference strain (strain due to inertial force). This differential strain always occurs on either the dorsal or ventral surface of the haltere, where the sensilla are located. Hence, it is hypothesized that the differential strain stimulates the sensilla and the location of the sensilla on the dorsal and ventral surfaces is in the context of the gyroscopic strain distribution.

### 6.2. Significance of the Haltere's Asymmetry

Based on the analytical and finite element estimation of the stress data, it is hypothesizes that “the haltere's asymmetry is correlated with the sensillum location on the dorsal and ventral surfaces” and can be explained as follows. Firstly, in the case of the haltere model with solid cross-section, the location of the maximum stress is at the thinnest cross-section of the stalk. From mechanics, it is known that any cantilever beam undergoes the maximum bending stress at the base. If at all the campaniform sensilla sense the maximum stress caused due to the out-of-plane bending deformation of the haltere, then they have to be located at the base. Since a solid cross-section throughout the length was considered, the section modulus is minimum at the thinnest cross-section and the bending stress is maximum at that location. However, the campaniform sensilla on both the dorsal and ventral surfaces are located somewhat away from the base.

Secondly, based on the haltere model with detailed cross-section at the stalk and base, the maximum stress occurs at a location in between the thinnest section and the base of the haltere. It can be argued that the haltere has variable cross-section throughout the length (hollow at the base, tubular cross-section with intermediate partitioning at the stalk, and solid cross-section at the knob). The variation in the cross-section leads to the minimum section modulus in between the base and the thinnest section rather than the thinnest cross-section. Therefore, it claimed that the sensilla have to be present at the section of where the section modulus is least and nature has designed the haltere in an asymmetric fashion in order to maximize the sensitivity of the campaniform sensilla.

## Figures and Tables

**Figure 1:** (a) A MEMS vibratory gyroscope (reproduced from [1]). (b) The first gyroscope developed by Draper Lab of MIT (courtesy of [2]).

**Figure 2:** (a) A picture of a soldier fly showing the head, thorax, abdomen, wing, and haltere. (b) A closer view of the haltere. (c) SEM image of the haltere base.

**Figure 3:** SEM images of the (a) soldier fly's haltere and sensilla pattern at the (b) ventral and (c) dorsal surfaces of the haltere base.

**Figure 4:** Sensilla classification as per Pringle [7].

**Figure 5:** (a) A 3D picture of the fly showing the flapping and sensing planes. (b) The sweep angle of the haltere in the flapping plane.

**Figure 6:** Cross-section of the thorax along the haltere's flapping plane.

**Figure 7:** (a) Different rotations of the fly. (b) Position “*P*” of the haltere in the flapping plane (*xy*). (c) An approximate model of the haltere.

**Figure 8:** Strain distribution due to (a) the inertial force and (b) the combined effect of the inertial and Coriolis forces due to the 10 rad/sec pitch rotations.

**Figure 9:** Stress distribution due to pitch, yaw, and roll rotations across the cross-section of the haltere base during the upstroke and downstroke motions.

**Figure 10:** Stress distribution due to pitch, yaw, and roll rotations across the cross-section of the haltere base during the upstroke motion.

**Figure 11:** Image of the haltere along the (a) dorsal and (b) lateral sides.

**Figure 12:** Curve fitting along the line *L*_2_.

**Figure 13:** Stress variation along the length of the haltere. (a) Analytically calculated. (b) Calculated using FEM analysis considering solid cross-section.

**Figure 14:** Cross-sectional view of the haltere (a) at the knob, (b) at the stalk, and (c) at the base [14].

**Figure 15:** Stress variation obtained from the FE model with variable cross-section into account.

**Table 1:** Coriolis forces for the pitch, yaw, and roll rotations.

Rotation	Force
*X* (pitch)	*A*(cos*β*cos*θe*_*z*_ + sin*βe*_*r*_)
*Y* (yaw)	−*A*sin*θe*_*z*_
*Z* (roll)	*A*(sin*β*cos*θe*_*z*_ − cos*βe*_*r*_)

## Data Availability

No experimental data were used to support this study.
